The article "Research on Multiplayer Posture Estimation Technology of Sports Competition Video Based on Graph Neural Network Algorithm" was published in 2022. Journal: Comput Intell Neurosci.

# Research on Multiplayer Posture Estimation Technology of Sports Competition Video Based on Graph Neural Network Algorithm

**DOI:** 10.1155/2022/4727375

**Published:** 2022-04-01

**Authors:** Xiaoping Guo

**Affiliations:** Shaanxi Normal University, Xi'an, Shaanxi 710000, China

## Abstract

With the explosive growth of the number of sports videos, the traditional sports video analysis method based on manual annotation has been difficult to meet the growing demand because of its high cost and many limitations. The traditional model is usually based on the target detection algorithm of manual features, and the detection of human posture features is not accurate. Compared with global image features such as line features, texture features and structure features, local image features have the characteristics of rich quantity in the image, low correlation between features, and will not affect the detection and matching of other features due to the disappearance of some features in the case of occlusion. Referring to the practice of Deep-ID network considering both local and global features, this paper adjusts the traditional neural network, and combines the improved neural network with the human joint model to form a human pose detection method based on graph neural network, and then applies the algorithm to multiperson human pose estimation. The results of several groups of comparative experiments show that the algorithm can better estimate the human posture in sports competition video, and has a good performance in solving multiperson pose estimation in sports game video.

## 1. Introduction

With the development of society, more and more sports videos have entered people's daily life. Analyzing these sports videos can not only bring more wonderful content to the audience but also find out the shortcomings of athletes for improvement. Accurate athlete detection and pose estimation are important links in sports video analysis. The existing human target detection and pose estimation algorithms have achieved good performance in general human detection tasks, but they will detect athletes and spectators at the same time in sports video, so they cannot further distinguish athletes' targets, which will interfere with the subsequent video analysis. At the same time, the sports video data with human body annotation is scarce, and the cost of obtaining a model suitable for the field of sports video is high. Athletes are a special case of general human body detection task. If the general human body detection model can be used to detect and estimate athletes in sports video, it can undoubtedly save a lot of cost. The analysis and understanding of sports video have a huge market demand [1], and can provide standard teaching cases for sports lovers. In addition, the statistics of various data of athletes in the video can not only help athletes improve their technical level, but also adjust the tactical deployment for the whole team, and help coaches and athletes improve the strength of the team to a certain extent. The demand for sports video analysis and understanding is increasing.

The existing target detection and human pose estimation technologies have achieved good performance in the general scene detection task based on pictures, but there are few algorithms and data for target detection in sports video scenes. The usual approach is to label these data, and then train the target detection algorithm with new data to obtain the detection model [2]. Although this method can achieve results, it needs to retrain the model every time, which requires a lot of labeling cost and training cost. There are many kinds of sports videos, and a video contains a large number of pictures [3], so it is undoubtedly expensive to label the video. When analyzing sports video, the focus is on athletes. The target detector trained based on general target detection task itself has the ability to recognize people. Similarly, human posture estimation for sports video is also one of many human posture estimation scenes. The human posture detector based on general scene training also has the ability to recognize human posture in sports video. Ifmmc1 the trained general detector can be directly used for the detection of athletes, it can undoubtedly greatly reduce the cost [4]. However, in sports video, people are crowded, occlusion often occurs between people, motion blur is serious, and the general target detector does not have the ability to distinguish ordinary spectators and athletes [5], which brings challenges to the use of general detector in sports video scenes.

This paper mainly studies the athlete detection and human posture estimation in sports video. Based on graph neural network algorithm and human posture estimation algorithm, combined with the characteristics of sports video, the target detection and human posture estimation model based on general data set training is transferred to the field of sports video, The purpose is to reduce the training and labeling cost of athlete detection and pose estimation for sports video, and improve the performance of athlete detection and human pose estimation in sports video. In this paper, the task of athlete detection and human posture estimation for sports video mainly focuses on the problem of multiperson motion in video. The LSP data set with 14 labeled joint points is adopted to meet the characteristics of multiperson motion and recognizable posture. The performance of this algorithm is compared with four mainstream methods of human pose estimation in multiple databases to verify the effectiveness of this algorithm in the field of multiperson pose estimation.

## 2. Related Work

Target detection is a basic task in the field of computer vision, and has always been a hot research topic. Before the introduction of depth neural network, the target detection algorithm is mainly realized by extracting the manual features of the image for feature matching [6]. Many image manual features such as sift and surf have achieved good results. A lot of work has tried to design different manual features for target detection according to the characteristics of detection targets, such as V-J detection, hog detection [7], and DPM [8] algorithm. The target detection algorithm based on manual features mainly uses the information of target color, texture and edge structure to recognize objects. It can achieve good results in a relatively simple background. However, in practice, the background changes in different fields are complex, and the image is often affected by illumination and resolution, resulting in target deformation and blur, so it is difficult to cover all the cases by manual features. The generalization ability of target detection algorithm based on manual features is weak. Therefore, the performance in complex scenes is not very good.

With the development of deep learning, human pose estimation algorithm based on deep learning has become the mainstream. The human posture estimation algorithm based on deep learning regards human posture detection as a key point regression problem, trains through a large number of data with joint point category and position annotation, and finally obtains a model that can predict the position and category of human joint points [9]. In the early days, people mainly studied single person pose estimation, that is, there is only one human body in the detected picture. The single person Newell et al. [10] designed an hourglass like network structure for attitude detection, and added a supervision signal in the middle of the network. The single person pose task only detects one human pose, which has simple picture background and less interference. The existing single person pose estimation algorithms have achieved good performance and achieved an accuracy of more than 93% on the single person pose estimation data set MPII. However, in practice, most pictures have multiple human bodies, so the single person pose estimation algorithm is no longer applicable. Compared with single person pictures, multiperson pictures have complex background and serious interference between people. The attitude estimation algorithm for multiperson faces more problems [11]. The existing multiperson attitude estimation algorithms are mainly divided into two categories: top-down multiperson attitude estimation algorithm and bottom-up multiperson attitude estimation algorithm. The top-down multiperson attitude estimation algorithm first detects the human body in the figure through target detection, then cuts out a single human body according to the detection frame and sends it to the single person attitude detector to obtain the human body attitude, and finally puts the single person's attitude back to the corresponding position in the original figure to obtain the human body attitude of all people [12]. Alphapose [13] algorithm introduces the spatial transformer network module to optimize the positioning accuracy of the detection frame and achieve a more accurate multiperson attitude estimation effect. Chen et al. [14] designed a cascaded pyramid network to complete multiperson attitude estimation through multiple regression and adjustment. The top-down multiperson attitude estimation algorithm decomposes the multiperson attitude detection problem into multiple single person attitude detection problems, which is realized by target detection and single person attitude detection. This method is simple and effective, but its performance will be affected by the target detection results. Because of the limitations of the target detection frame, when there are multiple people gathering and occlusion, there will be multiple human bodies in the target detection frame. At this time, the effect of the top-down multiperson pose estimation algorithm will be affected.

To sum up, the existing target detection algorithms are mainly based on convolutional neural network [15], and have achieved good performance on the general target detection data set. At the same time, the algorithm needs a lot of data-driven, and the cost of training a new model is high [16]. When target detection is carried out in some specific fields, the existing methods usually design and retrain the target detection model based on the data in this field. Although it can achieve good performance, it costs a lot. However, in practice, the specific target to be detected is often a specific example of a certain class in the general target detection task, such as van detection and athlete detection, which are special cases of vehicle detection and human body detection in the general target detection task. At this time, if the trained general target detection model can be used to detect these specific targets, it can not only reduce the training cost, but also improve the application scope of the general detection model. The existing algorithms pay more attention to how to improve the detection performance in specific fields, and there is less research on how to migrate the general target detection model to specific fields to achieve specific targets.

## 3. Multiperson Pose Estimation Algorithm Based on Graph Neural Network

### 3.1. Graph Neural Network Algorithm

The structure of neural network mainly includes convolution layer and pooling layer. The function of convolution layer is to extract abstract features by convolution kernel and reduce the number of parameters by local perception and weight sharing. The function of the pool layer is to aggregate and count the feature map extracted from the convolution layer, and further reduce the number of neurons by down sampling [17]. When using convolution check sample image block to extract abstract features, different regions of the sample image are treated equally, but in fact, the joint is only located in the central region of the positive sample image, so the central region plays a greater role in identifying the joint than other regions. Therefore, when extracting features, we should pay more attention to the central region and weaken the edge region. Therefore, this paper improves the convolution operation of neural network, and assigns different weights to the convolution operation in different regions of the image. Due to the similarity of the same species, although the appearance features of the same joint image block of different human bodies will be different due to different body shapes and postures, the difference is not very large, especially in the central area of the image, so they have similar local features. Since the same joint image blocks of different human bodies have similar local features, their global features will also have great similarity. The global features can also play a certain role in identifying joints. Therefore, in identifying joints, we should consider not only the local features of the image, but also the global features. Therefore, this paper improves the structure of the traditional neural network by referring to the deep id network in the face recognition algorithm, which considers both local and global features, and the global and local features of the image were extracted and combined as image features. The image features include 32-dimensional local features and 1-dimensional global features, which are mainly determined by local features, as shown in Figure 1.

Firstly, the local response of the color image is normalized to improve the generalization ability of the neural network. According to the size of the input vector and the global features of the output one-dimensional image, the neural network structure set in this paper is shown in Table 1, including 3 convolution layers, 4 pooling layers, 1 lead-in layer and 3 full connection layers. Some of the parameters are shown in Table 1.

The improved graph neural network contains three convolution layers. The meaning of the parameters of each convolution layer in Table 1 is similar. For example, the output parameter of convolution layer 3 is 9 × 9 × 32, where 32 is the number of convolution kernels. A convolution kernel corresponds to a feature extraction method. After convolution, a feature map is obtained, 9 × 9 represents the size of the characteristic image obtained after convolution, and the convolution step of all convolution layers is 1 × 1. The convolution layer activation function adopts the modified linear unit (ReLU) with strong anti-overfitting ability. ReLU will make the output of some neurons 0, which leads to the sparsity of the network, reduces the interdependence of parameters and alleviates the over fitting problem.

The learning algorithm of the improved CNN adopts the random gradient descent algorithm, and the objective function is set as

(1) $$\begin{array}{c} O\left(W\right)=\sum_{i=1}^{N}\left(f^{i}\left(W\right)-d^{i}\right), \end{array}$$

where *N* is the number of samples, *f*^*i*^(*W*) is CNN output, *d*^*i*^ is the sample classification label, and positive and negative samples are 1 and 0 respectively. The improved graph neural network contains three full connection layers, and the neurons in the layer are connected with all the neurons in the upper layer. In front of the full connection layer is the introduction layer, but the convolution layer 3 and the pooling layer 4 are introduced into the full connection layer. The activation function of the first two fully connected layers adopts the modified linear unit (ReLU), and the fully connected layer 3 adopts the logistic regression function, and the output is the joint label.

### 3.2. Human Pose Estimation of Single Frame Image

In this section, the video is divided into a series of single frame images. For each frame image, the position of each joint point of the upper body of the human body is obtained, and the posterior edge probability distribution of the wrist is calculated. Maximum likelihood estimation can be understood as a map estimator when the prior probability is uniformly distributed, and obtains the point estimation of the difficult to observe quantity according to the empirical data. The maximum a posteriori estimation is integrated into the prior distribution of the quantity to be estimated, which can be regarded as the regularized maximum likelihood estimation. In order to realize the human body pose estimation of a single frame image, the most commonly used graph structure model is used to represent the basic human body architecture, and the reasoning algorithm is used to obtain the exact joint position by transmitting messages between the parent node and the child joint point.

Figure 2 shows a schematic diagram of a structural model. The structure of human body is described by undirected graph G(E, *V*), where the vertex *v*_*i*_ ∈ *V* represents a human body part, and the edge line *e* represents the adjacent joint point *vi* and *vj* For example, in the human body structure, there is a physical connection between the left wrist and the left elbow. Use the human body configuration *P* = {*p*^1^, *p*^2^, ... *p^i^*, *p*^*n*−1^, *p^n^*} to describe the posture of the human body, where *p*^*i*^ =(*x*^*i*^,  *y*^*i*^, *θ*^*i*^) is used to describe the human body part *vi*.(*xi*, *yi*) represents the coordinates of the center point of the rectangular box of part *v*^*i*^, *θ*^*i*^ Indicates component *v*_*i*_ The direction of the rectangle. Given a frame of image *I*, the human body configuration *P* is defined as

(2) $$\begin{array}{c} P=k\cdot e^{\sum \varphi \left(p^{i},p^{j}\right)+\sum \phi \left(p^{i},I\right)},\;\left(i,j\right)\in E,\;i\in V, \end{array}$$

where *φ*(·) and Φ(·) are potential energy functions. Paired term potential energy function *φ*(*p*^*i*^, *p*^*j*^) model the geometric constraint relationship between two adjacent joint points by encoding the human body a priori model. Φ(*p*^*i*^, *I*) indicates the feasibility that the component *v*_*i*_ is located at the *p*^*i*^ position in the image *I*.

The best posture of human body in a single frame image is obtained by formula (1). Generally, the graph structure model has a tree structure, so two different reasoning algorithms can be used in reasoning. When reasoning with the maximum a posteriori (map), select the maximum product method to obtain the globally optimal maximum a posteriori estimation and the sum product method to obtain the edge distribution of the wrist, and take the edge distribution of the wrist as the a posteriori distribution probability of the tracking algorithm in the next stage.

In order to process video sequences more effectively, each frame needs to be read. Processing video frames mainly applies some processing functions to each video frame. As shown in Figure 3, the data processing module first divides the input sports video into frames, and unifies the size of the video frame to 1000 × 600 pixels, then detect people in each frame of the video based on the general target detector, then input the detection results obtained by the general target detector into the trained example feature metric classifier to obtain the athlete's detection results, and then fuse the multi frame detection results based on the video time domain context to obtain the optimized athlete's detection results.

### 3.3. Graph Neural Network Structure Model for Multiperson Attitude Estimation

In order to ensure the recall rate of athletes, this paper takes all the detection frames of the general target detector as candidate frames when the threshold is 0. Extracting the features of the detection frame is to extract the features of the image content contained in the detection frame. The CNN network in the detection model has extracted the features of the whole image. According to the position of the detection frame, the ROIAlign method is used to extract the features of the detection frame.

Firstly, the feature map is resized to the size of the original map by bilinear interpolation, and then crop is performed on the feature map according to the position of the detection frame. Then, the detection frame feature map max pool to a unified size. Finally, the detection frame feature map is linearly expanded to obtain one-dimensional detection frame features. The size of the feature map of the detection frame after Max pooling will change according to different convolution neural networks, so that the feature length of the one-dimensional detection frame is between 1024 and 2048. In particular, a two-stage target detection network with RPN structure, such as fast RCNN, will extract features from each detection frame for classification and frame regression, that is, each detection frame obtained by fast RCNN target detection algorithm has a unique depth feature corresponding to it. RPN network compares the predicted results with the real results, reflects the gap between the predicted and the real value through the user-defined “distance,” and optimizes the “distance” through the optimization algorithm, so the prediction is closer to the real value. In this paper, these features are directly used to identify the candidate frame as the feature of the candidate frame, The frame feature dimension extracted by the fast RCNN model used in this paper is 2048 dimensions.

The multilevel feature diagram is shown in Figure 4. To identify athletes, that is to distinguish athletes and nonathletes, the essence is to classify them according to the characteristics of candidate boxes. A feature vector *q* is defined to represent athletes, so that the candidate frame features of athletes are close to *Q* and the candidate frame features of nonathletes are far from Q. in this way, a threshold can be set to distinguish athletes from nonathletes.

From the candidate frame selection and feature extraction module, the 2048 dimensional depth feature corresponding to each detection frame can be obtained. This feature can be used to distinguish different detection frames, but cannot distinguish athletes from nonmobilization. Therefore, it is necessary to carry out a linear transformation on these features. This linear transformation module transforms the 2048 dimensional candidate frame feature into a 512 dimensional new feature. Initialize a 512 dimensional feature vector *Q* to represent the athlete. By continuously optimizing the parameters of this linear transformation module, the similarity between the new features of the athlete candidate box and *Q* becomes larger, and the similarity between the new features of the nonathlete candidate box and *Q* becomes smaller. The calculation formula of the linear transformation module is: *R* = tanh (*Wf*).

where *f* represents the original 2048 dimensional feature of the candidate box, *R* represents the 512 dimensional new feature after linear transformation, tanh is one of hyperbolic functions, and tanh () is hyperbolic tangent. In mathematics, the hyperbolic tangent “tanh” is derived from the hyperbolic sine and hyperbolic cosine of the basic hyperbolic function, and *W* is the weight parameter of the linear transformation module.

Firstly, initialize a 512 dimensional feature vector *Q* to represent the athlete, then select the candidate box and extract the features of the picture to obtain *n* 2048 dimensional candidate Box feature vectors F, and then linearly transform the candidate box features to have the same dimension as the athlete features to obtain *n* 512 dimensional candidate box features R. Then calculate the cosine similarity between each candidate frame feature *R* and athlete feature *Q* to obtain AI, where I represents the number of candidate frames, and the values are 1 to *n*. All the detection frames in a picture are regarded as a package, and the maximum cosine similarity between the candidate frame feature and the athlete feature is taken as the similarity S between the package and the athlete feature. Suppose *Q* represents an athlete, *R* represents a picture containing an athlete, then the positive packet similarity can be expressed as *s* (Q, R), P represents a picture without an athlete, and the negative packet similarity can be expressed as *s* (Q, P). Theoretically, the similarity between a picture containing an athlete and an athlete category is greater than a picture without an athlete, that is, *s* (Q, R) > *s* (Q, P).

The graph neural network is mainly composed of feature extraction layer, region recommendation layer, region of interest pooling layer and classification layer. Feature extraction layer and region recommendation layer have an important impact on the realization of network functions.  Figure 5 is the network structure diagram of the neural network, which integrates the functions of feature extraction, candidate box selection, location refinement and classification into the same network. The designed structure corresponds to the feature extraction layer, region recommendation layer, region of interest pooling layer and classification layer respectively.

Given a natural image containing human posture, its size P ∗ Q needs to be reduced to a fixed size M ∗ N and then input into the graph neural network. M ∗ N images first pass through the feature extraction layer in the network, use this layer to extract the feature map describing human posture, and share the feature map describing human posture image in the subsequent region suggestion layer and region of interest pooling layer. The part of the graph neural network that is only directly connected with the feature extraction layer is called the region recommendation layer, which can be used to generate candidate frames of human parts. The region suggestion layer first generates rectangular boxes of different sizes through the convolution layer, then uses the classification function to judge whether the image block contained in the generated rectangular box is a human body part or a background pixel, and simultaneously calculates the offset of the generated rectangular box to fine tune the position of the generated rectangular box. So far, the graph neural network has completed the positioning function of human parts. Considering that the region suggestion layer generates a rectangular box with non-fixed size, which cannot be directly used as the input of the classification layer, the region of interest pooling layer is introduced into the graph neural network. The region of interest pooling layer takes the original feature map and the generated rectangular box as the input at the same time, and extracts the feature vector of the image block in the generated rectangular box by blocking in the original human posture feature map, so as to ensure the output of the feature vector of fixed size. Finally, the fixed size feature vector is input to the classification layer, and the specific human body part type of the image block contained in the generated rectangular box is output.

Supervised learning is a machine learning task to infer a function from the marked training data. The training data includes a set of training examples. In supervised learning, Each instance consists of an input object (usually a vector) and a desired output value (also known as supervised signal) composition. Supervised learning algorithm is the function of analyzing the training data and generating an inference, which can be used to map new instances. An optimal scheme will allow the algorithm to correctly determine the class labels of those invisible instances. This requires that the learning algorithm is in a “reasonable.” The way is formed from a training data to an invisible situation. Before training the network, the position of each part of the human body is marked in a rectangular box to realize the supervised learning of network parameters. When testing the network, the static image containing human body is directly input. After the graph neural network, the image with a series of rectangular detection boxes and the fractional probability vector corresponding to the rectangular detection box are output.

### 3.4. Evaluating Indicator

The athlete detection and evaluation is the same as the evaluation standard of general target detection. This paper evaluates by calculating the joint sum intersection ratio IoU (interaction over union) between the detection result frame and the marked frame. When IoU >0.5, it is considered that the athlete is correctly detected.

For the estimation and evaluation of athletes' posture, there are two evaluation methods of human joint points: PCK [18] (percentage of correct keypoints) and OKS [19] (object keypoint similarity). This paper selects the commonly used OKS method, which will calculate the similarity between the two postures and give a score between 0 and 1. In this paper, the OKS scores of predicted posture and real posture are calculated. The OKs score is calculated as follows:

(3) $$\begin{array}{c} {\text{OKS}}_{p}=\frac{\sum_{i}\exp-d_{pi}^{2}/2S_{p}^{2}\sigma_{i}^{2}\delta \left(v_{pi}=1\right)}{\sum_{i}\delta \left(v_{pi}=1\right)}. \end{array}$$

*p* represents the ID of the person in the growth truth, and *i* represents the ID of the keypoint. *D*_*pi*_ represents the Euclidean distance between each person in the growth truth and the predicted key point of each person. *S*_*p*_ represents the scale factor of the current person, which is equal to the square root of the area occupied by the person in the ground truth. *σ*_*i*_ represents the normalization factor of the *i*-th bone point. Therefore, this is obtained by calculating the standard deviation of all ground truths in the data set, reflecting the standard deviation when labeling the current bone point. *v*_*pi*_ represents whether the *i*-th key point of the *p*-th person is visible. *δ* function for selecting visible points for calculation. When OKS >0.5, it is considered that the athlete's posture is correctly detected. Athlete detection and posture estimation are both kinds of detection tasks. According to the evaluation method of detection tasks, this paper selects three common evaluation indexes, namely maximum recall rate, AP value and P-R curve, which are defined as follows. For the test results, there may be four situations between the predicted value and the actual value: TP, FP, FN, TN. TP and FP respectively indicate that the predicted positive sample and negative sample are true, FN and TN respectively indicate that the predicted positive sample and negative sample are false. Where P in the P-R curve represents precision and *R* represents recall. The formula are as follows:

(4) $$\begin{array}{c} P=TP{\left(TP+FP\right)}^{-1},\\ R=TP{\left(TP+FN\right)}^{-1}. \end{array}$$

By setting different detection confidence thresholds, different detection results will be generated. The accuracy and recall rate of the detection results of each threshold can be calculated. The recall rate obtained by setting the confidence threshold to the minimum is the maximum recall rate. Calculate the accuracy and recall for each confidence threshold, and then take the recall as the abscissa and the accuracy as the ordinate to draw the P-R curve, which can well reflect the performance change of the detector. The AP value of target detection can be obtained by calculating the integral of the curve in the interval [0, 1]. The AP value is an important index to measure the performance of target detection. The larger the AP value, the better the performance of the detector.

This article selects two objective evaluation criteria to objectively evaluate the experimental results of this algorithm, one is the percentage of detected joints (PDJ) and the other is the percentage of correct parts (PCP). The specific meaning of PDJ evaluation standard is that for each joint point, when the distance between the predicted position and the real position (calculated by Euclidean distance here) is less than the given threshold, the joint point is correctly located. The PDJ value of each joint point changes with the change of threshold value. The resulting curve depicts the change trend of joint point positioning accuracy, which is called PDJ curve. The specific meaning of PCP evaluation standard is that when the two joint points corresponding to both ends of a human part are correctly positioned, the part is correctly positioned.

## 4. Experiment and Analysis

### 4.1. Experimental Setup and Data Set

Based on the video time domain context, the effective fusion of the detection results of different video frames can effectively improve the recall rate of athlete detection, and solve the problem of missing detection caused by motion blur to a certain extent, but it may also bring the risk of false detection. The optimization strategy of detection results based on time-domain context involves multiple super parameters. In order to ensure the optimization effect, these super parameters need to be set reasonably. The super parameters and value ranges involved are as follows: the value range of adjacent frame interval *n* is [0, 30], the value range of interframe similarity threshold *s* is [0, 64], the value range of local similarity threshold *D* is [0, 64], and the value range of supplementary detection frame confidence threshold *T* is [−1, 1]. In this paper, the grid parameter search method is used to experiment on NBA basketball video data set to determine the best parameter combination. In order to improve the efficiency of grid parameter search, the computational cost of parameter search can be reduced by removing some obviously unreasonable parameter ranges. According to experience, the search interval and search step of each super parameter are as follows: the search range of adjacent frame interval *n* is [0, 10], the search step is 1, the search range of interframe similarity threshold *s* is [0, 10], the search step is 1, the search range of local similarity threshold *D* is [0, 10], the search step is 1, the search range of supplementary detection frame confidence threshold *T* is [0, 1], and the search step is 0.1. After continuous parameter search, when the super parameters *N* = 3, *s* = 5, *d* = 2, *t* = 0.3, the sports competition video data set constructed in this paper can achieve good results. Parameter W represents the weight vector in the multilevel graph structure model. The process is as follows:

(5) $$\begin{array}{c} \underset{w}{\min}\langle \omega_{ij},w_{ij}\rangle +\sum C\max\left[0,1-y_{n}\langle w,\Phi \left(I^{n},l^{n},t^{n}\right)\rangle \right],\;y_{n}\in \left\{0,1\right\}. \end{array}$$

In the above formula, Φ(*n*) is the sparse feature of the n-th training image.

In this paper, the grid parameter search method is used to experiment on the data set to determine the best parameter combination. Grid search method is an exhaustive search method to specify parameter values. The optimal learning algorithm is obtained by optimizing the parameters of the estimation function through cross validation. That is, the possible values of various parameters are arranged and combined, and all possible combination results are listed to generate a “grid.” Then each combination is used for SVM training, and the performance is evaluated by cross validation. After the fitting function tries all the parameter combinations, it returns an appropriate classifier and automatically adjusts to the best parameter combination. In order to improve the efficiency of grid parameter search, the computational cost of parameter search can be reduced by removing some obviously unreasonable parameter ranges. According to experience, the search interval and search step of each super parameter are as follows: the search range of adjacent frame interval *n* is [0, 10], the search step is 1, the search range of inter frame similarity threshold *s* is [0, 10], the search step is 1, the search range of local similarity threshold *D* is [0, 10], the search step is 1, the search range of supplementary detection frame confidence threshold *T* is [0, 1], and the search step is 0.1.

At present, the mainstream human posture data sets used in the research include 2D and 3D. The 2D human posture data sets are shown in Table 2, BBG, and common data sets include MSCOCO, MPII, LSP, FLIC, posetrack and AI challenger.

Leeds sports pose is a sports pose data set, which is divided into sports, badminton, baseball, gymnastics, parkour, football, volleyball and tennis. It contains about 2000 pose notes, and the images are from the athletes of Flickr. Each image is a 3-channel color image, and each image is marked with 14 joint positions, and the left and right joints are always marked with human center. The LSP data set is collected from different motion scenes. Its extended version includes 11000 training samples and 1000 test samples. There are 14 labeled joint point types in the LSP data set, and the LSP data set does not need to be cropped, because the author of the data set provides preprocessed images. In the experiment, only the provided images need to be scaled to a fixed size. Therefore, the human posture estimation data set LSP is selected in this experiment, and other data sets such as FLIC, MSCOCO and Buffy pose are also used for comparison.

### 4.2. Evaluation of Multiperson Attitude Estimation Model

Figure 6 shows the loss curve during the training of the three-dimensional attitude estimation network. The training process is 300 rounds in total. It can be seen that the loss function (loss) value shows a decreasing trend with the increase of the number of training rounds, and tends to be stable after 250 rounds, indicating that the model training is gradually convergent.

We use a graph neural network algorithm for multiperson human pose estimation. The human posture estimation process is divided into two stages: detection component and positioning component [20]. In the first stage, the specific deep learning network is used as the human part detector to realize the detection function of human parts; In the second stage, a new spatial constraint relationship of human parts is designed to uniquely determine the position of each part from the candidate box of human parts, realize the positioning function of joint points, and finally complete the estimation process of human posture. In order to objectively verify the role of the component detection model based on graph neural network and the designed human component spatial constraint model in the whole algorithm, experiments on controlling a single variable are carried out on FLIC and Buffy databases, which can represent the overall performance of the traditional attitude estimation method. Green curve is the average PDJ curve obtained by hiding the spatial constraint model of human parts and directly taking the rectangular box position corresponding to the highest score probability vector output by fast R-CNN as the positioning result of human parts; The red curve is the average PDJ curve obtained by the algorithm. Comparing the green curve and purple curve longitudinally, it can be concluded that compared with the traditional methods, only using deep learning network to solve the problem of human posture estimation from the perspective of target detection has great advantages in positioning accuracy. In addition, as can be seen from Figure 7, both the component detection model based on fast R-CNN and the proposed human component spatial constraint model contribute to the final realization of accurate human pose estimation results.

In order to test the running time of this algorithm in the process of 3D human body pose estimation, this algorithm is compared with literature [20] and literature [21] under the same software and hardware conditions. The results are shown in Figure 7. The average time per frame of algorithm [20] is 32.801 s, because the model mainly matches the SMPL model with two-dimensional joint points based on parameter optimization, and the optimization process takes a lot of time; SMPL needs to consider not only the basic human body configuration, but also whether the joint density can control the movement of points. Therefore, when there are no obvious joints in the chest, several joints are added, while the number of joints on the hand is less. For better manikin expression, SMPL adds more points to finer parts, such as fingers. According to the area of normal people, there should be fewer points, but this is unfavorable to SMPL model. The average time per frame of algorithm [21] is 6.281 s. The model combines a large number of 3D attitude prior constraints and 2D data sets, so its attitude estimation has high efficiency; The average running time of each frame of the algorithm in this paper is 1.115 s, in which the process of two-dimensional human posture estimation takes an average of 0.015 s, and the process of three-dimensional SMPL model parameter estimation and three-dimensional joint point calculation takes an average of 1.10 s. The fully connected network structure design proposed in this paper saves a lot of model calculation time, improves the accuracy and maintains high efficiency.

### 4.3. Results of Comparative Experiments

In order to further illustrate the effectiveness of the algorithm in the field of human posture tracking, the performance of the algorithm is compared with four methods in videopose2.0 and VIPs Videopose databases. The four mainstream methods selected include: (1) the improved method of graph model in document [21], (2) the model proposed in document [22], (3) the extensible model proposed by document [23], and (4) the hybrid component model proposed in document [24]. In order to ensure the comparability of the experimental results, the training or test of the above four methods are exactly the same as that of the algorithm.

Generally speaking, the PDJ and PCP values of each algorithm when detecting the head are basically close to the real values, so the positioning results of these two joint points are not recorded in this experiment. This experiment only counts the positioning accuracy of 6 joint points and 4 parts (upper and lower arms) on videopose 2.0 and VIPs videopose databases.  Figure 8 shows the PDJ curve of this algorithm and the above four methods on VIPs Videopose database. As can be seen from Figure 8, the algorithm adopted in this paper is higher than the conventional algorithm in the positioning accuracy of each joint point, and can obtain better human posture tracking effect. In particular, for the wrist joint points most concerned in the process of human posture estimation, the positioning accuracy of this algorithm is significantly higher than that of the other four methods. For example, taking 30 pixels as the threshold, the wrist PDJ value of this algorithm is 98.3%, which far exceeds the PDJ value of reference [20] 82.1%, reference [21] 84.1%, reference [22] 78.2% and reference [23] 80.1%.

Table 3 shows the comparison results of PCP values of this algorithm and the above four methods (with 30 pixels as the threshold) on VIPs Videopose database. The PCP value of the waist of this algorithm is 95.9%, which far exceeds the PCP value of 63.8% in reference [20], 83.0% in reference [21], 92.5% in reference [22] and 81.0% in reference [23]. It is confirmed that the algorithm still maintains good positioning accuracy on VIPs videopose.

## 5. Conclusion

In this study, the structure of traditional neural network is improved. In order to study the posture estimation of multiple people in sports competition video, a human posture estimation algorithm based on graph neural network is adopted by using Multi level characteristic diagram. After statistics of 6 joint points and 4 parts on VIPs videopose database show that the graph neural network algorithm can complete the positioning function of human parts, so as to achieve accurate human body tracking effect. Comparing the PDJ curves and PCP values of varIoUs algorithms, it can be seen that the algorithm based on graph neural network greatly improves the positioning accuracy of varIoUs parts of the human body compared with other algorithms. Therefore, when applied to athlete posture tracking in sports competition video, this method can effectively estimate the posture of multiple people.

## Figures and Tables

**Figure 1:** Improved graph neural network structure.

**Figure 2:** Structural model of human upper body diagram.

**Figure 3:** Data processing module.

**Figure 4:** Multilevel characteristic diagram of athletes in sports competition.

**Figure 5:** Neural network structure diagram of human posture in sports video.

**Figure 6:** Loss curve of human posture estimation network.

**Figure 7:** Running time comparison of human pose estimate.

**Figure 8:** PDJ curve comparing this algorithm with other algorithms on VIPS-VideoPose database.

**Table 1:** Figure structural parameters of neural network.

Layer	Conv1	Pool1	Conv2	Pool2	Conv3
Input	64 ∗ 64 ∗ 3	60 ∗ 60 ∗ 32	30 ∗ 30 ∗ 32	24 ∗ 24 ∗ 32	12 ∗ 12 ∗ 32
Output	60 ∗ 60 ∗ 32	30 ∗ 30 ∗ 32	24 ∗ 24 ∗ 32	12 ∗ 12 ∗ 32	9 ∗ 9 ∗ 32
Size	5 ∗ 5 ∗ 3	2 ∗ 2 ∗ 1	5 ∗ 5 ∗ 32	2 ∗ 2 ∗ 1	5 ∗ 5 ∗ 32
Layer	Pool3	Pool4	FC1	FC2	FC3
Input	9 ∗ 9 ∗ 32	5 ∗ 5 ∗ 32	1 ∗ 1 ∗ 2400	1 ∗ 1 ∗ 2400	1 ∗ 1 ∗ 500
Output	5 ∗ 5 ∗ 32	1 ∗ 1 ∗ 32	1 ∗ 1 ∗ 2400	1 ∗ 1 ∗ 500	1 ∗ 1 ∗ 100
Size	2 ∗ 2 ∗ 1	5 ∗ 5 ∗ 1	—	—	—

**Table 2:** Human pose estimate datasets.

Dataset	Feature
LSP	The data comes from sports category labels, image zoom, only annotated in each picture-one person, 14 key points
FLIC	Data comes from hollywood movies, 10 key points
MPII human pose	The data comes from YouTube videos, which covers 410 human activities, each image has an activity tag, and 16 key points
MSCOCO	The data comes from the internet, it contains various activities, 17 key points
Al challenge	The data is captured from the internet. It is currently the largest human pose image data set, and 14 key point
PoseTrack	The data comes from the MPII human pose data set and 15 key points
Buffy	The data comes from a TV show. Line segments are provided to indicate the location, and the size and direction of the body parts are also provided

**Table 3:** Comparison of PCP value results between this algorithm and other algorithms on vipsvediopose.

Methods	Algorithm (%) [20]	Algorithm (%) [21]	Algorithm (%) [22]	Algorithm (%) [23]	Ours (%)
Neck	78.1	62.8	78.2	57.8	87.1
Elbow	80.9	69.3	79.4	54.7	88.2
Shoulder	91.7	83.3	90.5	34.2	95.1
Wrist	65.4	84.2	93.2	78.5	92.7
Waist	63.8	83.0	92.5	81.0	95.9

## Data Availability

The data used to support the findings of this study are available from the corresponding author upon request.
